RETRACTED

# Silencing of Long Non-coding RNA HOTTIP Reduces Inflammation in Rheumatoid Arthritis by Demethylation of SFRP1

**DOI:** 10.1016/j.omtn.2019.11.015

**Published:** 2019-11-26

**Authors:** Xumin Hu, Jianhua Tang, Xuyun Hu, Peng Bao, Weixi Deng, Jionglin Wu, Yuwei Liang, Zhipeng Chen, Liangbin Gao, Yong Tang

**Affiliations:** 1 Department of Orthopedics, Sun Yat-Sen Memorial Hospital, Sun Yat-Sen University, Guangzhou 510120, P.R. China; 2 Department of Spinal Surgery, Meizhou People’s Hospital, Meizhou 514031, P.R. China; 3 Center for Medical Genetics, Beijing Children’s Hospital, Capital Medical University, National Center for Children’s Health, Beijing 100045, P.R. China; 4 Medical Department, Sun Yat-Sen Memorial Hospital, Sun Yat-Sen University, Guangzhou 510120, P.R. China; 5 Guangdong Provincial Key Laboratory of Malignant Tumor Epigenetics and Gene Regulation, Sun Yat-Sen Memorial Hospital, Sun Yat-Sen University, Guangzhou 510120, P.R. China; 6 Department of Orthopedics, The First Affiliated Hospital of Sun Yat-Sen University, Guangzhou 510080, P.R. China

**Keywords:** rheumatoid arthritis, long non-coding RNA, HOTTIP, SFRP1, Dnmt3b, promoter methylation, Wnt signaling pathway

## Abstract

Accumulating evidence suggests long non-coding RNAs (lncRNAs) play crucial roles in the pathogenesis of rheumatoid arthritis (RA). Here, we aimed to define the role of HOXA transcript at the distal tip (HOTTIP) in RA pathogenesis in relation to SFRP1 methylation and Wnt signaling pathway. HOTTIP was found highly expressed, and SFRP1 was hypermethylated in RA synovial fibroblasts (RASFs). Next, gain- or loss-of-function experiments were conducted in RASFs to explore the effects of HOTTIP on the biological behaviors of RASFs. Silencing of HOTTIP or overexpression of SFRP1 inhibited RASF proliferation, invasion, and migration, while enhancing apoptosis. The relationship among HOTTIP, SFRP1, and Dnmt3b was determined using methylation-specific PCR (MSP), bisulfite sequencing PCR (BSP), RNA pull-down, RNA immunoprecipitation (RIP), and chromatin immunoprecipitation (ChIP) assays. The regulatory mechanisms of HOTTIP/Dnmt3b/SFRP1 were explored by altering their expression in RASFs. It was noted that HOTTIP could induce SFRP1 promoter methylation through recruitment of Dnmt3b and activate the Wnt signaling pathway. Finally, a rat RA model was established in order to evaluate the *in vivo* effects of HOTTIP and SFRP1, which suggested that HOTTIP silencing or SFRP1 elevation inhibited the progression of RA *in vivo*. Our key findings demonstrate the anti-inflammatory ability of HOTTIP silencing in RA through SFRP1 promoter demethylation. These findings support HOTTIP as a candidate anti-arthritis target.

RETRACTED

## Introduction

As a chronic inflammatory autoimmune disorder, rheumatoid arthritis (RA) leads to chronic inflammation of synovial tissues in joints, which can progress to irreversible joint destruction.^1^ RA is characterized by a plethora of symptoms, including synovial hyperplasia, joint swelling, pain, articular inflammation, and invasion, as well as cartilage and synovial membrane injury.^2^^,^^3^ Multiple risk factors, which include dyslipidemia, insulin resistance, obesity, diabetes, prednisone exposure, hypertension, inflammation, genetic variants, and physical inactivity, have been associated with the occurrence and progression of RA.^4^, ^5^, ^6^ Though early intervention with anti-inflammatory drug therapy improves the quality of life and clinical outcomes in patients with RA, the biological processes underpinning the pathogenesis of RA remain unclear.^7^^,^^8^ Understanding the underlying molecular mechanisms of the pathogenesis of RA can pinpoint new molecular targets for therapeutic development.^9^ Such research can aid the pursuit of successful clinical remission of RA via novel therapies.

Long non-coding RNAs (lncRNAs), a group of non-protein-coding transcripts longer than 200 nt, play crucial roles in the development of many diseases.^10^ lncRNAs modulate gene expression by binding to chromatin regulators and interfering with RNAs and thus exert downstream effects on cellular responses.^11^^,^^12^ HOXA transcript at the distal tip (HOTTIP) is a type of lncRNA capable of influencing various cellular processes, such as inhibition of cellular growth and promotion of apoptosis.^13^ In particular, HOTTIP has been identified as a key regulator lncRNA in the pathogenesis of knee osteoarthritis (OA).^14^ Furthermore, downregulation of HOTTIP was shown to impact cartilage integrity by upregulating integrin-α1 or DNA methyltransferase 3b (Dnmt3b) in OA.^15^ The possible role played by HOTTIP in RA has not been studied, suggesting a need to explore its potential involvement. Secreted Frizzled-related proteins (SFRPs), commonly known as Wnt inhibitors, have the ability to bind extracellularly to Wnts.^16^ SFRP1 has been associated with inflammatory responses and found to be downregulated in RA synovial fibroblasts (RASFs).^17^ Additionally, the downregulation of SFRP1 caused by promoter hypermethylation was linked to the induced keloid development by activating the Wnt/β-catenin signaling pathway and decreasing Dnmt1.^18^

In the present study, we aimed to explore the function of HOTTIP in the pathogenesis of RA and its underlying mechanisms. We have proved that HOTTIP, SFRP1, and the Wnt signaling pathway cooperated with each other to regulate the proliferation and apoptosis of RASFs, as well as inflammatory responses in RA.

RETRACTED

## Results

### Silencing of HOTTIP Inhibits Proliferation and Promotes Apoptosis of RASFs in RA

First, the lncATLAS website (http://lncatlas.crg.eu/) predicted that HOTTIP was mainly located in the nucleus (Figure S1). Upregulation of HOTTIP is reported in OA, and it is involved in the progress of OA.^15^ However, the role of HOTTIP in RA has not been studied, so we wanted to explore whether HOTTIP was involved in the progression of RA and compared the expression of HOTTIP in OA and that in RA. As further determined by qRT-PCR, the HOTTIP expression in synovial tissues from patients with RA was remarkably higher than in synovial tissues from patients with OA (Figure 1A; p < 0.05). The RASFs and OA synovial fibroblasts (OASFs) were further isolated from the synovial tissues from patients with RA and OA, and the isolated primary cells were identified by determining vimentin expression using immunocytochemical staining (left panel, Figure 1B). Both fluorescence *in situ* hybridization (FISH) and RNA quantitation after nuclear and cytoplasmic fractionation showed that HOTTIP was mainly localized in the nucleus of RASFs (Figures 1B and 1C), suggesting that the dysregulation of HOTTIP may be involved in the functions of RASFs. Thereafter, HOTTIP was successfully overexpressed or silenced in RASFs and OASFs using lentivirus infection (Figure 1D). The migratory potential of activated RASFs can affect at least partly joint destruction and the spread of destructive arthritis between joints.^19^^,^^20^ The behaviors of RASFs were then evaluated using a water-soluble tetrazolium salt-1 (WST-1) assay, Transwell assay, scratch test, and flow cytometry. The results provided evidence that silencing of HOTTIP led to markedly reduced cell proliferation (Figure 1E), invasion (Figure 1F) and migration abilities (Figure 1G), and induced cell apoptosis (Figure 1H). On the contrary, overexpression of HOTTIP accelerated the proliferation, migration and invasion abilities, and hindered apoptosis of RASFs (Figures 1E–1H).

**Figure 1:** Downregulation of HOTTIP Suppressed the Proliferation and Enhanced the Apoptosis of RASFs (A) The HOTTIP expression in RASFs and OASFs determined by qRT-PCR. (B) Immunocytochemical staining of vimentin expression in the isolated of RASFs and OASFs (×200) and subcellular localization of HOTTIP in RASFs and OASFs by FISH (×400). (C) Subcellular localization of HOTTIP in RASFs determined by qRT-PCR after nuclear and cytoplasmic fractionation. (D) The infection efficiency of lentivirus expressing overexpressed (oe)-HOTTIP or short hairpin RNA (sh)-HOTTIP in RASFs was determined by qRT-PCR. GAPDH was used as an internal control. (E–H) Cell proliferation, invasion, migration (×200), and apoptosis were assessed in RASFs upon overexpression or silencing of HOTTIP determined by WST-1 assay (E), Transwell assay (F), scratch test (G), and flow cytometry (H), respectively. *p < 0.05 compared with RASFs infected with lentivirus expressing oe-negative control (NC); ^#^p < 0.05 compared with RASFs infected with lentivirus expressing sh-NC. The results were expressed as mean ± SD. Comparisons between two groups were conducted by means of t test. The data at different time points (E) were analyzed by repeated-measurement ANOVA. Comparisons among multiple groups were analyzed by one-way ANOVA. The experiment was repeated three times.

RETRACTED

### Restoration of SFRP1 Inhibits Migration and Promotes Apoptosis of RASFs

SFRP1 has been previously implicated in the regulation of RA,^17^^,^^21^ but few reports explained the mechanism of SFRP1 involved in the regulation of RA. In order to further explore the significance of SFRP1 in RA, we determined the expression of SFRP1 in RASFs and OASFs by qRT-PCR and that in synovial tissues of patients with RA and OA by immunohistochemical staining. It was observed that SFRP1 was expressed at a lower level in RASFs and synovial tissues of patients with RA than in OASFs or synovial tissues of patients with OA (Figures 2A and 2B). It has been previously revealed that promoter methylation of SFRP1 enhanced tumor progression in renal cell carcinoma.^22^ Cytosine phosphate guanine (CpG) islands were predicted in the promoter region of SFRP1 (http://www.urogene.org/cgi-bin/methprimer/Methprimer.cgi) (Figure S2). Hence, we tested the methylation of SFRP1 in the promoter region by methylation-specific PCR (MSP) assay. Furthermore, we treated RASFs by aza-2′-deoxycytidine (Aza-dC) to block the activity of methyltransferase, and mRNA expression of SFRP1 was subsequently determined by qRT-PCR. MSP assay revealed that SFRP1 was hypermethylated in RASFs cells and the methylation level of SFRP1 in OASFs was remarkably lower than that in RASFs (Figure 2C). Moreover, the mRNA expression of SFRP1 in RASFs increased notably after 0.5 mmol/L Aza-dC treatment for 34 h (Figure 2D). Next, SFRP1 was overexpressed in RASFs in order to explore its modulatory effects on the biological functions of RASFs. The data obtained from WST-1 assay, Transwell assay, scratch test, and flow cytometry, overexpression of SFRP1 led to a decrease in proliferation (Figure 2E), invasion (Figure 2F), and migration (Figure 2G) and increased apoptosis of RASFs (Figure 2H). Taken together, our findings indicated that SFRP1 was hypermethylated in RASFs, which reduced SFRP1 expression, and the restoration of its expression suppressed the invasive and migratory potentials of RASFs.

RETRACTED

**Figure 2:** Overexpression of SFRP1 Suppressed Proliferation and Enhanced Apoptosis of RASFs (A) The SFRP1 expression in RASFs and OASFs determined by qRT-PCR. GAPDH was used as an internal control. (B) SFRP1 expression in the synovial tissues of patients with RA and OA detected by immunohistochemical staining (×400). The synovial tissue sections of patients with RA were used as positive control. (C) Methylation of SFRP1 promoter region predicted through the bioinformatics website and identified by MSP assay (H_2_O, double-negative control; IVD, methylation-positive control; NL, unmethylated positive control; U, unmethylation; M, methylation). (D) SFRP1 expression in Aza-dC-treated RASFs detected by qRT-PCR. (E–H) Proliferation, invasion (×200), migration, and apoptosis of RASFs were assessed upon overexpression of SFRP1 by means of WST-1 (E), Transwell assay (F), scratch test (G), and flow cytometry (H), respectively. **p < 0.05 compared with OASFs; *p < 0.05 compared with RASFs infected with lentivirus expressing oe-NC; ^#^p < 0.05 compared with RASFs treated with DMSO. The results were expressed as mean ± SD. Comparisons between two groups were conducted by means of t test. The experiment was repeated three times.

### HOTTIP Inhibits SFRP1 by Inducing Promoter Methylation of SFRP1 by Recruiting Dnmt3b

HOTTIP was predicted to bind to SFRP1 promoter using the website Long Target (http://lncrna.smu.edu.cn/show/DNATriplex) (Figure S3). To further explore the regulatory relationship between HOTTIP and SFRP1, the expression of SFRP1 in RASFs infected with lentivirus expressing overexpressed (oe-HOTTIP) or short hairpin RNA (sh-HOTTIP) was determined by qRT-PCR and western blot analysis. Consequently, HOTTIP was found to negatively regulate the expression of SFRP1 (Figure 3A; p < 0.05). However, SFRP1 could not affect HOTTIP expression (Figure 3B). It was shown that HOTTIP may downregulate SFRP1 expression and thus affect cell cellular functions.

**Figure 3:** Binding of HOTTIP to Dnmt3b Promoted Promoter Methylation of SFRP1 and Downregulated the Expression of SFRP1 (A) The SFRP1 expression in RASFs determined by qRT-PCR and western blot analysis after HOTTIP was overexpressed or silenced. (B) HOTTIP expression in RASFs determined by qRT-PCR after SFRP1 was overexpressed or silenced. (C) SFRP1 promoter methylation analyzed by MSP (H_2_O, double negative control; IVD, methylation positive control; NL, unmethylated positive control; U, unmethylation; M, methylation). (D) SFRP1 promoter methylation analyzed by BSP, respectively (black circle, methylation site; white circle, unmethylated site; blank group refers to RASFs without treatment). (E) The expression of SFRP1 in RASFs overexpressing HOTTIP treated with Aza-dC. (F) Enrichment of three DNA methyltransferases (Dnmt1, Dnmt3a, Dnmt3b) in the SFRP1 promoter region and enrichment of Dnmt3b in the SFRP1 promoter region after silencing of HOTTIP. (G) The presence of HOTTIP co-immunoprecipitated with Dnmt3b from RIP assay. (H) The binding relationship between Dnmt3b and HOTTIP identified by RNA pull-down assay. *p < 0.05 compared with RASFs infected with lentivirus expressing oe-NC; ^#^p < 0.05 compared with RASFs infected with lentivirus expressing sh-NC. **p < 0.01 compared with RASFs treated with Aza-dC; ^##^p < 0.01 compared with immunoglobulin G. The results were expressed as mean ± SD. Comparisons between two groups were conducted by means of t test. Comparisons among multiple groups were analyzed by one-way ANOVA. The experiment was repeated three times.

RETRACTED

In a RA rat model, the methyltransferase Dnmt1 was found to bind to SFRP1 promoter methylation to promote the progression of RA.^23^ We thus speculated that HOTTIP may affect the occurrence of RA by regulating SFRP1 promoter methylation. The MSP results showed that overexpression of HOTTIP positively regulated the promoter methylation of SFRP1 (Figure 3C). Bisulfite sequencing PCR (BSP) results showed that the promoter methylation of SFRP1 was induced by overexpression of HOTTIP and inhibited when HOTTIP was silenced in RASFs (Figure 3D). The addition of Aza-dC was found to attenuate the decrease in SFRP1 induced by HOTTIP overexpression (Figure 3E). These results suggested that the silencing of HOTTIP could regulate the transcriptional and promoter methylation levels of SFRP1 and restore the transcription of SFRP1 to a certain extent by inhibiting the activity of methyltransferase. The enrichment of three methyltransferases (Dnmt1, Dnmt3a, and Dnmt3b) relative to IgG was detected by chromatin immunoprecipitation (ChIP) assay, and results showed that, compared with Dnmt1 and Dnmt3a, the enrichment of Dnmt3b in the SFRP1 promoter region was remarkably increased, suggesting that Dnmt3b was mainly enriched in the SFRP1 promoter region. Moreover, the silencing of HOTTIP attenuated the enrichment of Dnmt3b in the SFRP1 promoter region (Figure 3F). RNA immunoprecipitation (RIP) results showed that following extraction of RNA from coimmunoprecipitated protein solution, the presence of HOTTIP in RNA co-immunoprecipitated with Dnmt3b antibody, as detected by qRT-PCR (Figure 3G). Next, RNA pull-down assay further verified that Dnmt3b could bind to HOTTIP (Figure 3H). Taken together, these observations demonstrated that lncRNA HOTTIP could interact with Dnmt3b and recruit Dnmt3b to the SFRP1 promoter region, resulting in hypermethylation of the CpG islands and inhibition of SFRP1 transcription.

RETRACTED

### HOTTIP Activates the Wnt Signaling Pathway and Induces Inflammatory Responses in RASFs by Binding to Dnmt3b

Since we have proved that HOTTIP downregulated SFRP1 expression by promoting the promoter methylation of SFRP1 through recruiting Dnmt3b, and it was earlier reported that SFRP1 was an inhibitor of Wnt signaling pathway.^24^^,^^25^ So, we further investigated whether the Wnt signaling pathway was involved in the functions of RASFs mediated by HOTTIP.

Western blot analysis and qRT-PCR revealed that silencing of HOTTIP inhibited mRNA and protein expression of key genes of the Wnt signaling pathway (β-catenin, C-myc, CCND1), while overexpression of HOTTIP increased these mRNA and protein expression of key genes of the Wnt signaling pathway (β-catenin, C-myc, CCND1) (Figure 4A). Further, the sh-Dnmt3b and oe-Dnmt3b vectors were constructed to silence and restore Dnmt3b expression, respectively. The expression of SFRP1 was elevated upon silencing of Dnmt3b and was reduced upon overexpression of Dnmt3b (Figure 4B). Additionally, silencing Dnmt3b and overexpressing HOTTIP together significantly reduced SFRP1 expression (Figure 4C). Next, the expression of key genes of the Wnt signaling pathway (β-catenin, C-myc, CCND1), inflammatory factors (interleukin-6 [IL-6], IL-8), and RA marker genes (fibronectin and MMP3) was further determined when Dnmt3b expression was altered. The findings indicated that overexpression of Dnmt3b elevated the expression of β-catenin, C-myc, and CCND1, while sh-Dnmt3b reduced their expression. In contrast, further overexpression of HOTTIP in cells harboring silencing Dnmt3b could significantly inhibit the expression of β-catenin, C-myc, and CCND1 (Figure 4D). The expression of inflammatory factors (IL-6, IL-8) and RA marker genes (fibronectin and MMP3) was consistent with that shown in Figure 4F, while the expression of aforementioned factors was reduced upon silencing Dnmt3b (Figures 4D–4F). These results demonstrated that HOTTIP could activate the Wnt signaling pathway by mediating Dnmt3b and thereby promote inflammatory responses.

**Figure 4:** HOTTIP Inhibited SFRP1 by Recruiting Dnmt3b, Thereby Activating the Wnt Signaling Pathway and Suppressing the Inflammatory Response of RASFs (A) The mRNA and protein expression of key genes of the Wnt signaling pathway in response to overexpression or silencing of HOTTIP, as determined by qRT-PCR and western blot analysis. (B) The expression of Dnmt3b in RASFs transduced with sh-Dnmt3b or oe-Dnmt3b, as determined by qRT-PCR. RASFs were infected with lentivirus expressing sh-Dnmt3b or oe-Dnmt3b in the presence of HOTTIP for the subsequent experiments. (C) The mRNA and protein expression of SFRP1 in RASFs determined by qRT-PCR and western blot analysis. (D) The mRNA and protein expression of key genes of the Wnt signaling pathway in RASFs determined by qRT-PCR and western blot analysis. (E) Levels of inflammatory factors in RASFs measured by ELISA. (F) The mRNA and protein expression of RA marker genes in RASFs determined by qRT-PCR and western blot analysis. GAPDH was used as internal control. *p < 0.05 compared with RASFs infected with lentivirus expressing oe-NC; ^#^p < 0.05 compared with RASFs infected with lentivirus expressing sh-NC; & p < 0.05 compared with RASFs infected with lentivirus expressing sh-Dnmt3b. The results were expressed as mean ± SD. Comparisons between multiple groups were performed using one-way ANOVA. The experiment was repeated three times.

RETRACTED

### Silencing of HOTTIP Inhibits the Progression of RA by Upregulating SFRP1 *In Vivo*

The rat model of RA was identified by observing paw swelling and pathological changes in the lesions. H&E staining showed ankle impairment in the rats after modeling, with inflammatory cells and synovial cells enriched in the joint clearance (Figures S4A and S4B). To study the effects of HOTTIP-mediated SFRP1 on the progression of RA *in vivo*, the production of inflammatory factors and the aggravation of RA were analyzed by conducting gain- and loss-of-function experiments. It was found that overexpressing HOTTIP or silencing SFRP1 exacerbated paw swelling in RA rats after 24 days of treatment, while silencing of HOTTIP or restoration of SFRP1 alleviated the paw swelling (Figure 5A). Moreover, rescue experiments suggested that the aggravated paw swelling induced by HOTTIP overexpression was inhibited by additional restoration of SFRP1 (Figure 5A). These results suggested that silencing of HOTTIP could prevent the progression of RA *in vivo* by upregulating SFRP1.

**Figure 5:** HOTTIP Enhanced Progression of RA by Suppressing SFRP1 *In Vivo* RA rats were injected with lentiviruses expressing sh-HOTTIP, sh-SFRP1, oe-HOTTIP, and/or oe-SFRP1. (A) Representative images and quantification of paw-swelling scores of rats on the 24^th^ day. (B) The pathological changes at rat joints detected by H&E staining (×200; scale bar, 50 μm). (C) Expression of β-catenin and C-myc in synovium of rats measured by immunohistochemical staining (×200; scale bar, 50 μm). The synovial tissue sections of patients with RA were used as positive controls. (D) Serum levels of inflammatory factors (IL-6 and IL-8) in rats measured by ELISA. (E) Expression of MMP3 in rats detected by immunofluorescence staining (×400; scale bar, 25 μm). *p < 0.01. The results were expressed as mean ± SD. Comparisons among multiple groups were analyzed by one-way ANOVA. n = 15.

RETRACTED

H&E staining displayed that the articular surfaces of the ankle joints in RA rats injected with lentivirus harboring oe-HOTTIP or sh-SFRP1 were destroyed, showing a lack of obvious joint space, significant synovial hyperplasia, and extensive infiltration of inflammatory cells, with a large number of inflammatory and synovial cells in the joint space. On the contrary, RA rats injected with lentivirus harboring sh-HOTTIP or oe-SFRP1 showed relatively complete articular surfaces, mild hyperplasia of synovial cells, and mild inflammatory cell infiltration. The infiltration of inflammatory cells aggravated by HOTTIP overexpression was reversed by additional restoration of SFRP1 (Figure 5B). These findings verified that HOTTIP could enhance the proliferation and infiltration of synovium in RA by regulating SFRP1 and thus aggravate the progression of RA. Next, immunohistochemical staining, ELISA, and immunofluorescence staining revealed that the expression of β-catenin and C-myc in the synovium (Figure 5C), the serum levels of IL-6 and IL-8 (Figure 5D), as well as expression of MMP3 (Figure 5E) in the synovial membrane of rats, all were markedly increased by upregulation of HOTTIP or silencing of SFRP1 in RA rats but decreased when HOTTIP was silenced or SFRP1 was overexpressed. Moreover, the upregulation of HOTTIP reversed the inhibitory effects of oe-SFRP1 on the expression of β-catenin and C-myc in synovium (Figure 5C), the serum levels of IL-6 and IL-8 (Figure 5D), as well as expression of MMP3 in the synovial membrane of rats (Figure 5E). The aforementioned data suggested that HOTTIP induced activation of the Wnt signaling pathway and promoted progression of RA by inhibiting SFRP1 *in vivo*.

## Discussion

In RA, excessive accumulation of cytokines and chemokines has been associated with persistent chronic inflammation and immune response.^26^ DNA methylation patterns and gene expression profiles of RA provide a new understanding of the occurrence and development of RA.^27^ In recent years, multiple lncRNAs have been demonstrated to participate in the progression of RA by regulating DNA methylation, as well as histones.^28^^,^^29^ This study provided evidence that silencing HOTTIP could inhibit SFRP1 promoter methylation and block the Wnt signaling pathway via the recruitment of Dnmt3b, which effectively inhibited the progression of RA.

RETRACTED

Based on our findings, HOTTIP was highly expressed in RASFs. Similarly, HOTTIP was found to be overexpressed in human pancreatic cancer.^30^ Another study demonstrated that HOTTIP was highly expressed in OA cartilage, which contributed to the progression of OA and endochondral ossification.^14^ Our study also indicated that inhibition of HOTTIP could inhibit the proliferation and enhance the apoptosis of RASFs. Consistently, a recent study suggested that knockdown of HOTTIP inhibited proliferation and induced apoptosis of hand synovial fibroblasts, which contributed to alleviated synovial hyperplasia and arthritis in RA.^31^ Similarly, silencing of HOTTIP has been found to suppress the progression of OA.^15^

We found that the loss of HOTTIP could inhibit inflammatory responses of RASFs and the progression of RA, as reflected by reduced levels of IL-6 and IL-8, MMP3, and fibronectin in RASFs upon silencing HOTTIP. It has been reported that diminished IL-6 and IL-1β levels are associated with suppressed cell proliferation and inflammatory responses in RA.^32^ Reduced levels of IL-6 and IL-8 have also been found to be correlated with the anti-inflammatory effect of heat shock protein 72 on RA.^33^ Moreover, MMP3 was induced in fibroblast-like synoviocytes of RA, which was correlated with the progression of RA.^34^ Bertoncelj et al. have similarly demonstrated that the silencing of HOTTIP in RA-inhibited inflammatory, proliferative, and adhesive properties of synovial fibroblasts by epigenetic mechanisms (M.F. Bertoncelj et al., 2017, AGU, abstract).

In addition, we showed that when SFRP1 promoter methylation was induced in RASFs, it lowered SFRP1 expression. Concordant with our finding, SFRP1 was found as poorly expressed in fibroblast-like synoviocytes of RA.^21^ Additionally, low expression of SFRP1 was also found in OA, where its upregulation attenuated cartilage degradation and chondrocyte hyperthrophic marks.^35^ lncRNAs are known to affect behaviors of cells by regulating a variety of target genes.^36^ In the present study, using BSP, MSP, RNA pull-down, RIP, and ChIP assays, we demonstrated that HOTTIP could interact with Dnmt3b and recruit Dnmt3b to SFRP1 promoter, which resulted in hypermethylation of the CpG islands and consequent inhibition of SFRP1 transcription. Upregulation of SFRP2 induced by 5-Aza-dC was found to suppress fibronectin production and proliferation and induce apoptosis of fibroblast-like synoviocytes by repressing SFRP2 promoter methylation via reduction of Dnmt1.^37^ Apart from embryogenesis and oncogenesis, SFRPs are known to be involved in the pathogenesis of RA by functioning as modulators of the Wnt signaling pathway.^38^ Similar to our findings, β-catenin, C-myc, and CCND1, the key genes of the canonical Wnt signaling pathway, were found inhibited in fibroblast-like synoviocytes upon upregulation of SFRP4, which in turn suppressed the progression of adjuvant arthritis.^39^ Others have reported that the inhibition of the Wnt/β-catenin signaling pathway caused by paricalcitol can ameliorate RA.^40^ In a previous study of osteosarcoma, the knockdown of HOTTIP was demonstrated similarly to suppress cell proliferation and promote cell apoptosis via inhibiting the Wnt/β-catenin signaling pathway.^41^ Together with our results, it appears evident that HOTTIP can inhibit SFRP1 and activate the Wnt signaling pathway by mediating Dnmt3b, thereby upregulating the levels of inflammatory factors and RA marker genes.

RETRACTED

In summary, the key findings of the study revealed that silencing of HOTTIP repressed SFRP1 promoter methylation and blocked the Wnt signaling pathway by decreasing Dnmt3b, thereby inhibiting proliferation and inflammatory responses and inducing apoptosis of RASFs (Figure 6). Thus, based on the current evidence, therapeutic strategies could be directed toward the downregulation of HOTTIP, which may comprise a potentially viable molecular target in the treatment of RA. Further studies are required, however, to fully understand the specific mechanisms by which HOTTIP may mediate other Wnt signaling pathway molecules and impact the pathology of RA.

**Figure 6:** HOTTIP Promotes SFRP1 Promoter Methylation by Recruiting Dnmt3b through Which HOTTIP Inhibits SFRP1 and Activates the Wnt Signaling Pathway, Thereby Inducing the Production of Inflammatory Factors and Enhancing the Proliferative and Migratory Abilities of RASFs

## Materials and Methods

### Ethical Statement

The study was conducted under the approval of the Ethics Committee of Sun Yat-Sen Memorial Hospital, Sun Yat-Sen University. All participating patients signed informed consent documentation. All experiments were conducted in strict accordance with the Helsinki Declaration. All animal experiments were ethically acceptable with the approval of the Animal Care and Use Committee of Sun Yat-Sen Memorial Hospital, Sun Yat-Sen University.

### Study Subjects

Synovial tissues were extracted from 28 patients with RA and 26 patients with OA diagnosed in Sun Yat-Sen Memorial Hospital, Sun Yat-Sen University, from January 2015 to December 2017. Among the enrolled RA patients, there were 16 females and 12 males, with a median age of 53.24 ± 4.54 years. OA patients included 15 females and 11 males, with a median age of 56.23 ± 3.16 years. No clinical heterogeneity was observed in the baseline characteristics of all cases. The diagnosis of the patients was in accordance with the 1987 RA classification criteria of the American College of Rheumatology (ACR). All the included patients had no injury of major organs or hematological diseases. Patients who met any of the following conditions were excluded: severe organ dysfunction, long-term history of Western medicine, advanced-stage deformity, or mental disorders.

RETRACTED

### Cell Isolation and Culture

Primary RASFs and OASFs were isolated from synovial tissues of patients with RA and OA by treatment with 1.5 mg/mL collagenase and 0.04% hyaluronidase as published previously.^17^^,^^42^ The isolated primary RASFs and OASFs were cultured in DMEM supplemented with 10% fetal bovine serum (FBS), 100 U/mL penicillin, and 100 μg/mL streptomycin at 37°C with 5% CO_2._ RASFs and OASFs at passage 4 were identified with antibody to vimentin on a flow cytometer. The cells were incubated with dimethyl sulfoxide (DMSO) containing 0.5 μmol/L methyltransferase inhibitor 5-Aza-dC (Zymo Research, Orange, CA, USA) for 24 h.

Lentiviruses were packaged using 293T cells with LV5-green fluorescent protein (GFP) vector (carrying transgene) or pSIH1-H1-copGFP vector (carrying short hairpin RNA [shRNA] for gene silencing). LV5-GFP vector carrying oe-HOTTIP, oe-Dnmt3b, oe-SFRP1, and oe-NC as well as pSIH1-H1-copGFP vector carrying shRNAs against HOTTIP (sh-HOTTIP), DNMT (sh-DNMT), SFRP1 (sh-SFRP1), or negative control shRNA (sh-NC) were synthetized by Shanghai Gene Pharma (Shanghai, China). RASFs in the logarithmic phase were infected with the aforementioned lentiviruses. The infection efficiency was quantified by measuring the expression of GFP observed under a fluorescence microscope at 48 h after infection.

### RNA Isolation and Quantitation

Total RNA was extracted using the Trizol method (Thermo Fisher Scientific, Waltham, MA, USA). RNA samples were treated with DNase to avoid genomic DNA contamination. Reverse transcription quantitative polymerase chain reaction (qRT-PCR) was carried out in accordance with the instructions of the Primescript RT reagent kit (TaKaRa Bio, Dalian, Liaoning, China) and the SYBR Premix Ex Taq II kit (Takara Bio, Shiga, Japan). The primers were synthesized by RiboBio (Guangzhou, Guangdong, China), as shown in Table 1. Fold changes were calculated by means of relative quantification (2^−ΔΔCt^ method).^43^

**Table 1:** Primer Sequences for qRT-PCR

Gene	Primer Sequence
HOTTIP	F, 5′-TACCGGAATAGTGCTGGGGA-3′
	R, 5′-TGCGTGCTGCTCTGAGTTTA-3′
SFRP1	F, 5′-ATGAGTGCCCCACCTTTCAG-3′
	R, 5′-AATGCTGCAAGAACAAGCCG-3′
β-catenin	F, 5′-TACCTCCCAAGTCCTGTATGAG-3′
	R, 5′-TGAGCAGCATCAAACTGTGTAG-3′
CCND1	F, 5′-AAAGAATTTGCACCCCGCTG-3′
	R, 5′-GACAGACAAAGCGTCCCTCA-3′
C-myc	F, 5′-GCCACGTCTCCACACATCAG-3′
	R, 5′-TCTTGGCAGCAGGATAGTCCTT-3′
Fibronectin	F, 5′-CCGTGGGCAACTCTGTC-3′
	R, 5′-TGCGGCAGTTGTCACAG-3′
MMP3	F, 5′-CGGTTCCGCCTGTCTCAAG-3′
	F, 5′-CGCCAAAAGTGCCTGTCTT-3′
GAPDH	F, 5′-CGGAGTCAACGGATTTGGTCGTAT-3′
	R, 5′-AGCCTTCTCCATGGTGGTGAAGAC-3′
Dnmt1	F, 5′-CGCATCCTTACCTCTGTCCC-3′
	R, 5′-ACCCCAGCATTTGCCGAATA-3′
Dnmt3a	F, 5′-GCCCTCCGGGTTTGAAAAGA-3′
	R, 5′-TCAGCATCTCCAGAACTCGG-3′
Dnmt3b	F, 5′-GGGAAGACTCGATCCTCGTC-3′
	R, 5′- CCGTCTCAGGGACTGTGTGT-3′

HOTTIP, HOXA transcript at the distal tip; SFRP1, secreted frizzled related protein 1; CCND1, cyclin D1; MMP3, matrix metalloproteinase-3; GAPDH, glyceraldehyde-3-phosphate dehydrogenase; Dnmt1, DNA methyltransferase 1; Dnmt3a, DNA methyltransferase 3a; Dnmt3b, DNA methyltransferase 3b; F, forward; R, reverse.

RETRACTED

### Western Blot Analysis

Total protein was extracted and separated by 10% sodium dodecyl sulfate-polyacrylamide gel electrophoresis (SDS-PAGE) (Millipore, Billerica, MA, USA). The proteins were then transferred to the polyvinylidene fluoride membrane, which was subsequently incubated with following primary antibodies: SFRP1 (ab4193, 1:230), Dnmt1 (ab19905, 1:100), Dnmt3a (ab4897, 1:1,000), Dnmt3b (ab79822, 1:1,000), β-catenin (ab16051, 1:400), CCND1 (ab134175, 1:10,000), C-myc (ab32072, 1:1,000), fibronectin (ab23750, 1:100), MMP3 (ab52915, 1:1,000), and glyceraldehyde-3-phosphate dehydrogenase (GAPDH; ab37168, 1:100) (all from Abcam, Cambridge, UK) overnight at 4°C. After that, horseradish peroxidase (HRP)-conjugated goat anti-rabbit secondary antibody (ab9482, 1:5,000, Abcam, Cambridge, UK) was incubated with the membranes at room temperature for 1 h. Next, the images of the membranes were obtained after reaction with enhanced chemiluminescence (Shanghai Baoman Biotechnology, Shanghai, China). Gel image analysis was performed using ImageJ software, and the ratio of the gray value of target protein band to that of GAPDH was calculated.

### FISH

FISH was used to detect the subcellular localization of HOTTIP in RASFs.^44^ Specifically, the cell slides were placed at the bottom of a 24-well plate, and the cells were seeded on slides in the plate at a density of 5 × 10^3^/well. After 24 h of culture, cells were washed with 1× phosphate-buffered saline (PBS). After being fixed with 4% paraformaldehyde for 10 min at room temperature, cells were penetrated with PBS containing 0.5% Triton X-100 and blocked with pre-hybridization solution at 37°C. The cells were incubated with hybridization solution containing HOTTIP probe overnight at 37°C. After 4′,6-diamidino-2-phenylindole (DAPI) staining for 30 min in dark, the slides were mounted. The cells were observed under a laser confocal microscope (ECLIPSE E800, Nikon, Tokyo, Japan).

RETRACTED

### Nuclear and Cytoplasmic Fractionation

Nuclear and cytoplasmic RNA fractions were separated according to the instructions of the PARIS kit (Life Technologies, Gaithersburg, MD, USA). The cells were collected and washed with PBS. After centrifugation at 500 × *g* for 5 min, the pellets were suspended in 500 μL cell fractionation buffer and incubated on ice for 5–10 min. After centrifugation at 500 × *g* for 5 min at 4°C, the supernatant (cytoplasmic fractions) was centrifuged in a 2-mL sterile enzyme-free tube at 500 × *g* for 5 min at 4°C. In addition, the pellets (nuclear fractions) were resuspended with 500 μL cell fractionation buffer and 500 μL 2× lysis/binding buffer. After the removal of the supernatant, pellets (nuclear fractions) were mixed with pre-cooled 500 μL cell fractionation buffer and 500 μL absolute ethanol and transferred to the adsorption column, which was put into a collection tube. The column containing 700 μL of reaction solution each time was centrifuged at 12,000 × *g* for 30 s. The column was washed twice with 500 μL washing buffer and eluted with 10 μL elution buffer at 12,000 × *g* for 30 s twice to obtain pure nuclear fractions. Nuclear and cytoplasmic expression of HOTTIP was determined by qRT-PCR with primer sequences shown in Table 2. 12S rRNA and GADPH served as the positive control of the cytoplasm, while U6 and 45S rRNA was the positive control of the nucleus.

**Table 2:** Primer Sequences for Nucleus and Cytoplasm Isolation

Gene	Primer Sequence
U6	F, 5′-CTCGCTTCGGCAGCACATATAC-3′
	R, 5′-AACGCTTCACGAATTTGCGTGTC-3′
12S rRNA	F, 5′-CGTAAAGCGTGTTAAAGCATCATACT-3′
	R, 5′-TGGGTCTTAGCTATGGTGTATCAG-3′
45S rRNA	F, 5′-GACACGCTGTCCTTTCCCTA-3′
	R, 5′-GTCTGACACGCAGCAAAGTC-3′

12S rRNA, 12S ribosomal RNA; 45S rRNA, 45S ribosomal RNA; F, forward; R, reverse.

### MSP

Genomic DNA was extracted from RASFs using a genomic DNA purification kit (QIAGEN, Hilden, Germany). Bisulfite modification of DNA was performed with the use of an Intergen CpGenome DNA modification kit (Intergen, New York, NY, USA), according to the manufacturer’s protocol. Un-methylated cytosine was converted to uracil by bisulfite, while methylated cytosine remained intact. MSP was performed using SFRP1 methylation-specific primers (Table 3). The PCR products were analyzed on a 3% Tris/borate/EDTA (TBE) agarose gel and subjected to image analysis using a gel imaging system.

**Table 3:** Primer Sequences for MSP and BSP

Gene	Primer Sequence
SFRP1(M)	F, 5′-AGTTTGGTTAATATGGTGAAATTTC-3′
	R, 5′-ACCTAAACTAAAATACAATAACGCT-3′
SFRP1(U)	F, 5′-TTTGGTTAATATGGTGAAATTTTGT-3′
	R, 5′-TACCTAAACTAAAATACAATAACACT-3′
BSP	F, 5′-GTTTGGGAGGTTAAGGTAGGAGTAT-3′
	R, 5′-ACAAACCCATAAAATTATAAAAACTTTTT-3′

SFRP1, secreted frizzled-related protein 1; BSP, bisulfite sequencing PCR; F, forward; R, reverse.

RETRACTED

### BSP

The PCR product was subjected to agarose gel electrophoresis. The recovery step was carried out in accordance with the specifications of the agarose gel DNA recovery kit (Tiangen Biotech, Beijing, China). The harvested DNA was cultured in Luria-Bertani (LB) solid medium containing X-gar, isopropyl-b-D-thiogalactopyrano-side (IPTG), and ampicillin in a shaker at 37°C. At least 10 single colonies (white clones) were selected. Colony PCR was performed using BcaBEST sequencing primers and methylation specificity universal primers. The positive recombinants were cultured overnight and then sequenced. The bisulfite sequencing primers are listed in Table 3.

### ChIP

ChIP was performed as described in the specifications of the EZ-Magna ChIP TMA kit (Millipore, Billerica, MA, USA). RASFs were cross-linked with 1% formaldehyde for 10 min and re-suspended in cell lysis buffer (150 mM NaCl, 50 mM Tris [pH 7.5], 5 mM EDTA, 0.005% NP40, 0.01% Triton X-100) containing protease inhibitors. Next, the cell lysate was sonicated to obtain chromatin fragments. 100-μL DNA fragments were added with 900 μL of ChIP dilution buffer and 20 μL of 50× protease inhibitor cocktail (PIC) and 60 μL of Protein A agarose/salmon sperm DNA. The DNA fragment was co-immunoprecipitated with the use of 1 μL rabbit antibodies to Dnmt3b (ab79822, 1:1,000), Dnmt1 (ab19905, 1:100), Dnmt3a (ab4897, 1:1,000) (all from Abcam) overnight. Rabbit anti-IgG (ab172730, Abcam) was added as NC. Each tube was added with 60 μL of protein A agarose/salmon sperm DNA for 2 h at 4°C. The DNA was eluted twice with 250 mL ChIP wash buffer. Finally, the eluted DNA was de-crosslinked. SFRP1 DNA promoter was quantified by qRT-PCR (Table 4).

**Table 4:** Primer Sequences of SFRP1 Promoter

Gene	Primer Sequence
SFRP1	F, 5′-AGCTGTTGTGCTGATACCGT-3′
	R, 5′-ACCAAGTCCATCACTCAGGC-3′

SFRP1, secreted frizzled-related protein 1; F, forward; R, reverse.

### RIP

A Magna RIP kit (Millipore, Bedford, MA, USA) was used for RIP. Cell lysate (100 μL) was incubated with magnetic beads pre-bound with rabbit antibody to Dnmt3b (ab79822, 1:1,000–1:5,000, Abcam) or normal mouse antibody to IgG at 4°C overnight. The immunoprecipitated complexes were centrifuged and washed with 500 μL of RIP wash buffer. After treatment with proteinase K, the immunoprecipitated RNA was isolated with Trizol-chloroform and subjected to qRT-PCR to detect the enrichment of HOTTIP.

### RNA Pull-Down Assay

HOTTIP RNA fragments were synthesized *in vitro* using T7 RNA polymerase (Ambion, Austin, TX, USA) and then purified using the RNeasy plus mini kit (QIAGEN, Hilden, Germany) and DNase I (QIAGEN, Hilden, Germany). HOTTIP RNA was biotinylated with a biotin RNA labeling kit (Ambion, Austin, TX, USA). The cell lysate was incubated with 400 ng biotinylated RNA and 500 μL RIP buffer for 1 h at room temperature, and a portion of the cell lysate was taken as input. The cell lysate was incubated with streptavidin-conjugated magnetic beads for 1 h at room temperature. The content of Dnmt3b protein was detected by western blot analysis.

RETRACTED

### Cell Proliferation Assay

In an aseptic environment, 100 μL suspension of RASFs (about 5,000–10,000 cells) was cultured in a 96-well plate at 37°C with 5% CO_2_ overnight and incubated with 10 μL WST-1 solution for 2 h. A cytotoxicity test was carried out with cells treated with Aza-dC (10 μL/well) at 37°C with 5% CO_2_ for 4 h, followed by an incubation with 10 μL WST-1 solution. The optical density (OD) values at 450 nm were detected with a spectrophotometer.

### Transwell Assay

A Matrigel-coated Transwell chamber (8 μm pore size; Corning, Tewksbury, MA, USA) was maintained with DMEM containing 20% FBS at 37°C for 1 h prior to assessment. At the 48^th^ h after transfection, the apical chamber was cultured with 100 μL RASF suspension (1 × 10^9^ cells/L) at 37°C with 5% CO_2_ for 24 h. After the non-invaded cells were removed with PBS washing, the cells in the chamber were fixed with 4% methanol. The cells stained with 0.1% crystal violet were counted under an inverted microscope and photographed. Migration distance and the number of invaded cells were quantified in five random fields of view.

### Scratch Test

Horizontal lines were evenly drawn across the well every 0.5–1 cm using a marker pen behind the 6-well plate (at least five lines per well). The cells (5 × 10^5^ cells/well) were cultured overnight. The cells were scratched perpendicular to the horizontal lines using a pipette. The cells were then washed three times with PBS and cultured with serum-free medium in a 37°C, 5% CO_2_ incubator, following the removal of debris. The scratches were photographed at the 0^th^ h and 36^th^ h under an inverted microscope.

### Flow Cytometry

RASFs at passages 3–6 were seeded into a 6-well plate and stained with 5 μL Annexin V-fluorescein isothiocyanate and propidium iodide at 4°C for 5 min under conditions void of light. Cell apoptosis was detected on FACSCanto II flow cytometer (BD Biosciences, San Jose, CA, USA) and analyzed using Diva software (BD Biosciences).^45^

### Immunocytochemistry

RASFs and OASFs at passage 5 were fixed, washed, and then treated with 3% H_2_O_2_ for 10 min. After PBS washing, the RASFs and OASFs were blocked with blocking solution for 15 min. Next, the RASFs and OASFs were probed with antibody to vimentin (1:100) overnight at 4°C, in accordance with the instructions of the kit (BPICC30-1KT, Hefei Protein Biotechnologies, Hefei, China). After development with diaminobenzidine, the RASFs and OASFs were observed and photographed under a microscope.

RETRACTED

### ELISA

The levels of inflammatory factors IL-6 and IL-8 were measured according to the instructions of an ELISA kit (Vafioskan Flash; Thermo Fisher Scientific, Waltham, MA, USA).^46^

### RA Model Establishment

120 Lewis rats aged 6–8 weeks and weighing 180–200 g were selected as experimental animals. First, 15 rats were randomly selected and left untreated as normal controls. The RA model was constructed in the remaining rats (n = 105) as outlined in a previous study.^47^ Lentiviruses expressing oe-NC, sh-NC, oe-HOTTIP, sh-HOTTIP, oe-SFRP1, sh-SFRP1, or both oe-HOTTIP and oe-SFRP1 were constructed and collected and were injected into Lewis rats as previously described.^48^ The day of the first injection was regarded as day 1. The hind paw thickness was measured, and the degree of RA was scored on day 24: 0–1 point = no detectable pathology (the appearance was normal with a flexible and evasive body, and the paw could support the body weight with highest grip strength); 1–2 points = arthritis onset (slight swelling of the joint above the paw); 2–4 points = mild arthritis (swollen joint with inflammation in the paw); 4–6 points = mild-to-moderate arthritis (swollen joint with last finger deformed inward; the paw could transiently support its body weight with decreased flexibility and grip strength); and 6–8 points = severe arthritis (severe joint, paw, and finger swelling, with deformation of joints and legs, lack of support in the upper part, loss of weight, lack of flexibility, no grip strength, climbing and eating affected).^42^ Rats were euthanized by intravenous injection of 3% pentobarbital sodium (P3761; Sigma-Aldrich, Milwaukee, WI, USA). The synovial tissues at the joints of rats were collected for immunohistochemical, immunofluorescence, and H&E staining assays.

### Immunohistochemical Staining

The synovial tissues were sectioned at 4 μm thickness and routinely dewaxed, followed by antigen retrieval by microwave heating. The sections were washed with PBS and then blocked with normal goat serum. The synovial tissue sections of patients with RA were used as positive controls. The synovial tissues were stained as outlined in the instructions of the Histostain SP-9000 kit (Zymed Laboratories, South San Francisco, CA, USA). Primary antibodies to β-catenin (ab16051, 1:400, Abcam) and C-myc (ab32072, 1:1,000, Abcam) were used for incubation. Five representative visual fields (direct optical microscopy, Nikon, Japan) were selected for observation, and the number of positive cells was counted.

RETRACTED

### Immunofluorescence Staining

Synovial tissues were fixed overnight in 4% paraformaldehyde and sliced into 4-μm-thick sections. The sections were penetrated and fixed with pre-cooled methanol for 15 min. The sections were blocked with 2% bovine serum albumin and 5% goat serum for 60 min. Immunofluorescence staining was performed with synovial tissues incubated with rabbit primary antibody to MMP3 (ab52915, 1:1,000, Abcam) at 4°C overnight and Cy3-labeled IgG (ab6939, Abcam) for 2 h at room temperature. The tissues were stained with 1 mg/mL DAPI. Images were captured on a Leica DMRA2 fluorescent microscope (Leica Microsystems, Bannockburn, IL, USA) using a Leica DC 500 camera. The numbers of fibronectin- and MMP3-positive cells were quantified using ImageJ software.

### H&E Staining

H&E staining was performed in order to observe pathological changes in joints.^49^ Paraffin-embedded tissues were sectioned into 5-μm-thick blocks. Tissue sections were stained with hematoxylin for 5–10 min. The sections were subsequently rinsed with tap water and blued using 1% aqueous hydrochloric acid. The sections were stained in eosin for 1–2 min. Synovial tissues were observed under an optical microscope. The image was captured by ImageJ image processing software.

### Statistical Analysis

All data were analyzed using SPSS 21.0 statistical software (IBM, Armonk, NY, USA). The experiments were repeated three times. Measurement data were expressed as mean ± SD. Comparisons between two groups were conducted by means of t test. Kolmogorov-Smirnov test was performed to assess normality of distribution and homogeneity of variance. Comparisons of measurement data conforming to the normal distribution and homogeneity of variance between two groups were performed by unpaired t test and those among multiple groups were assessed by one-way ANOVA with Tukey post-hoc tests. The data at different time points were analyzed by repeated-measurement ANOVA. p value < 0.05 was considered as statistical significance.

## Author Contributions

J.T., X.H., and L.G. designed the study. P.B. and X.H. collated the data. Z.C. and Y.T. carried out data analyses and produced the initial draft of the manuscript. W.D., J.W., and Y.L. contributed to drafting and polishing the manuscript. All authors read and approved the final manuscript.

## Conflicts of Interest

The authors declare no competing interests.

## Supplemental Information

Document S1. Figures S1–S4

Document S2. Article plus Supplemental Information
